# Low-cost commercial borosilicate glass slides for passive radiation dosimetry

**DOI:** 10.1371/journal.pone.0241550

**Published:** 2020-12-30

**Authors:** S. F. Abdul Sani, M. H. U. Othman, Amal Alqahtani, K. S. Almugren, F. H. Alkallas, D. A. Bradley

**Affiliations:** 1 Department of Physics, Faculty of Science, University of Malaya, Kuala Lumpur, Malaysia; 2 College of Medicine, University of Imam Abdulrahman Bin Faisal, Dammam, Saudi Arabia; 3 Department of Physics, Princess Nourah Bint Abdulrahman University, Riyadh, Saudi Arabia; 4 Centre for Biomedical Physics, Sunway University, Subang Jaya, Malaysia; University of Magdeburg, GERMANY

## Abstract

For x- and gamma- irradiations delivering entrance doses from 2- up to 1000 Gy to commercial 1.0 mm thick borosilicate glass microscope slides, study has been made of their thermoluminescence yield. With an effective atomic number of 10.6 (approximating bone equivalence), photon energy dependency is apparent in the low x-ray energy range, with interplay between the photoelectric effect and attenuation. As an example, over the examined dose range, at 120 kVp the photon sensitivity has been found to be some 5× that of ^60^Co gamma irradiations, also with repeatability to within ~1%. The glow-curves, taking the form of a single prominent broad peak, have been deconvolved yielding at best fit a total of five peaks, the associated activation energies and frequency factors also being obtained. The results indicate borosilicate glass slides to offer promising performance as a low-cost passive radiation dosimeter, with utility for both radiotherapy and industrial applications.

## 1. Introduction

One-dimensional (1-D) glass luminescence systems have been investigated by a number of researchers, accommodating a range of ionizing radiation dosimetry applications [1–4]. The glass matrix, manifestly amorphous silica (SiO_2_), occasionally shows evidence of local crystallite domains but is otherwise disordered. Such local micro-crystallite arrangements typically extend over only a relatively few lattice constants [5]. It has long been known that strain as well as extrinsic dopants and irradiation can modify the optical properties of such amorphous material, with vacancies and interstitial atoms created within the medium as a result of the various interactions. The typically non-crystalline structure glass is relatively resistant to radiation damage and thus has been widely used for purposes that include the encasement of radioactive material, even at highly elevated levels [6]. Encapsulation can range from use in radiation laboratory sources through to waste forms, previously including ejection to deep oceanic waters, a practice now eschewed.

Beyond the more typical scientific and kitchen glassware (Pyrex), borosilicates, have recently begun to find interest in thermoluminescnce (TL) dosimetry [7, 8]. The boronic content suggests potential for neutron TL dosimeters, with limited studies to-date [9]; similarly, Ge-doped silica neutron responses [10, 11]. The five main electron and hole traps identified in borosilicate glass compromise non-bridging oxygen centres (boron oxygen hole centres, BOHC), iron (II) and iron (III) centres, silica- and alkali-ions [12, 13]. Extending from this has been investigations of absorption of energy during irradiation. Electron/hole pairs generated and trapped during irradiation can be thermally stimulated leading to release of the stored energy as light, familiarly referred to as thermoluminescence. The light intensity is recorded as a function of sample temperature, producing one or more TL peaks, release at greater temperature equating to deeper trapping levels. Dosimetry applications favour TL emission intensity proportional to absorbed dose, calibration allowing determination of dose. TLD readers, manual and automatic, are widely available. For TL dosimeters used in personnel or environmental dosimetry, tissue-equivalence and high sensitivity are required. While satisfying some of these factors, the well-established phosphor forms (e.g. LIF:Mg,Ti) have several drawbacks, including a hygroscopic nature and relatively poor spatial resolution, typically of the order of a few mm, as well as cost. In such respect, commercial borosilicate glass would seem to offer features encouraging interest as competitor TLDs, including a softening point of 820°C, sufficiently low to suggest relative ease of fabrication if needed.

Present TLD work examines borosilicate glass in the form of microscope cover slips, exhibiting advantageous characteristics, including offering a ready-made mechanically robust product in various thicknesses, also being chemically inert, biocompatible, reusable and easily sterilizable. Due to the rich presence of intrinsic defects, x-ray irradiated borosilicate glass gives rise to appreciable TL [8]. In particular, for the penetrating photon irradiations of interest herein, the responses are characterized in terms of mass-dependent sensitivities, for radiation dose, dose-gradients and dose-rates of practical consequence in radiotherapy and radiation sterilization. Made from a mixture of silica and boric oxide (B_2_O_3_), it has an effective atomic number, Z_eff_, of 10.6, making it useful in bone dosimetry (as for example in potentially evaluating dose in the radiotherapy of bone sarcoma), albeit requiring more detailed account for soft-tissue dosimetry than TLD-100.

## 2. Experiment and methods

Commercial microscope glass slides (HmbG Chemicals, Germany) with thickness varying between 1.0 to 1.2 mm have been used for present investigations. Samples of these were prepared by cutting the glass into dimensions of approximately (0.5 × 0.5 × 0.1) ± 0.1 cm, use being made of a diamond cutter. The mass of each sample was measured using an electronic balance, allowing TL yields to be normalised to unit mass of the irradiated medium. Prior to irradiation the glass samples were annealed in a furnace at 400 °C, reducing exposure/triboluminescence history. To avoid surface abrasions and contamination, vacuum tweezers were used to handle the TL materials. Finally, to minimize light exposure pre- and post-irradiation, other than during readout the dosimeters were kept in darkened conditions. For TL sensitivity studies the dosimeters were irradiated to x- and gamma rays using sources located at the University of Malaya Department of Physics. An ERESCO 200 MF4 x-ray facility provided 120 kVp beams, delivering doses ranging from 2 to 10 Gy at a constant dose rate of 2.128 mGy/s. The X-ray tube output dose rates in air, obtained at the centre of the field (65.5 cm from the Al filter), was calibrated via use of an Raysafe Xi MAM R/F ionisation chamber. Gamma irradiations were carried out using a ^60^Co irradiator (mean energy 1250 keV) offering dose rate at the time of irradiation of 1.58 Gy/min, exposing the samples to doses in the two ranges 2- to 10 Gy and 250- to 1000 Gy. TL read-outs were obtained using a Harshaw Model TLD 3500 reader consisting of a photomultiplier tube (PMT) in light-tight containment and an Electrometer recording the PMT signal. WinREMS software provided for generation of the TL glow curves. The time-temperature profile (TTP) was obtained with a pre-heat temperature of 50°C, followed by a heating rate of 25°C/s and an acquisition time of 12 s. The maximum temperature was set to 350°C. The readings were made under a slow nitrogen gas flow, suppressing sample triboluminescence and oxidation, also reducing oxidation of the heating element and associated light emission. The delay between irradiation and readout was kept constant at 24 h, low temperature glow curve contributions reducing as a result of thermal fading at ambient temperatures.

## 3. Results and analysis

### 3.1. Dose response

Figs 1 and 2 show the TL response of x- and gamma-ray irradiated borosilicate glass, covering doses of 2–10 Gy and 0.2–1 kGy respectively. For the 120 kVp x-rays, the samples were located on the central axis of the x-ray source at a focus to surface distance of 68 cm. For both source irradiations the regression coefficient (R^2^) was greater than 0.98. The x-ray TL response (see Fig 1) was found to be of the order of 5× that of the gamma irradiations, a result of the greater absorption obtained at lower photon energies, unsurprising given the appreciable low-energy X-ray photoelectric cross-sections. Further apparent, with comparison now made of Figs 1 and 2, is that the initial strongly linear dose dependent behavior is maintained, with proportional sensitivity for the gamma-irradiated medium continuing through to the higher dose levels. Summarily, this can be described as a situation of high dynamic dose range, reflective of considerable utility. In practical use pre-determination of the dose dependence is essential for the specific TL material. In a previous ^60^Co borosilicate study [14], for doses from 150 mGy to 20 Gy, linear correlation of glow peak intensity to dose was also observed, determined for two low and high temperature dominant peaks, the former centred at some 120°C and the latter near 230°C. The observed variation in radiation sensitivity was related to trap filling, depletion and formation, occurring at different rates, also to low temperature peak instability and the differential in time taken to deliver the doses.

**Fig 1:** TL response for the 2 to 10 Gy dose range. Errors are standard error of the mean, with error bars typically smaller than the size of the data points.

**Fig 2:** TL response of gamma-irradiated borosilicate glass slides for doses from 0.2 to 1 kGy. Errors are standard error of the mean. (Note: the error bars are typically of the size of the data points).

The sensitivity of the samples can be linked to several factors. One should realize that the sensitivity is strongly dependent upon the type and concentration of dopants (activators) of the TL materials. It is well recognized that different batches of materials will have different TL sensitivities. The sensitivity, as defined before, depends largely upon the readout system used in the measurement as well as the annealing procedure applied to the TL medium. In addition, according to Furetta (2003) [15], the variations in TL sensitivities are mainly due to the variation in the mass of the detectors as well as contamination of sample surfaces. Study of the sensitivity has been reported by Bos (2001) [16] investigating dependence on the physical form of the TL materials, including mono- or poly-crystalline powder, sintered, thin and thick chips, all of which can affect the sensitivity of the TL materials. Apart from that, according to (Mckeever, 1995) [17], the sensitivity of TL materials can be influenced by the sensitivity of the photomultiplier tube (PMT) itself, the utilized heating rate as well as the intrinsic stability of the TLD readout system and the method of measurement of the system (glow peak area between two chosen temperatures, or the height of a particular peak). Other than that, the efficiency of light detection system such as the geometrical light collection efficiency, optical filter and the detector efficiency can also affect the TL sensitivities of the phosphor. As such, the sensitivity of borosilicate glass slides was calculated in units of TL yield.Gy^-1^.mg^-1^, investigated in accord with Eq 1 (as detailed by Furetta, 2003 [15]):

$$\text{Sensitivity}=\frac{TL\;Intensity}{Incident\;dose\;x\;mass\;of\;TL\;material}$$ (1)

Fig 3 shows this for doses from 2 Gy to 10 Gy. The sensitivity dependencies include the cross-sectional dimensions of the glass slides (reflected in normalization to sample mass) as well as the concentration of the various impurities and defects, boron included, potentially inhomogeneous within and across the samples. The decreasing trend with dose concerns the reducing availability of unfilled traps with increase in dose [18]. Nevertheless, at greater dose, a useable signal-to-noise ratio is retained [19].

**Fig 3:** Log plot of the TL sensitivity of borosilicate glass samples irradiated to doses ranging from 2 to 10 Gy.

### 3.2. Repeatability and linearity index

Repeatability has importance for dosimeter reuse. Fig 4(a) shows six randomly chosen sets of measurement, in use of 120 kVp x-rays the linear response reproducibility being better than 1%. An R^2^ of no less than 0.993 has been obtained up to six cycles. Fig 4(b) shows an enlarged view of TL yield for doses 2 and 10 Gy.

**Fig 4:** TL response for two 120 kVp irradiation cycles (a) for doses from 2- to 10 Gy; (b) enlarged view for doses 2- and 10 Gy for six repeat doses.

Further analysis of dose response has been carried out, use being made of the linearity index *f(D)* (normalised dose response), according to the formula (2) below (as detailed by Furetta, 2003 [15]):

$$f(D)=\frac{TL(D)/D}{TL(D_{1})/D_{1}}$$ (2)

with *TL(D)* the dose response at dose *D* and *D*_*1*_ the lowest dose at which the dose response is linear. Within this definition, *f(D)* > 1, *f(D)* = 1 and *f(D)* <1 imply supralinearity, linearity and sublinearity respectively. Fig 5 indicates that while a quasi-linear response is obtained for the 120 kVp x-ray irradiations, for the much more energetic ^60^Co gamma irradiation over the same 2- to 10 Gy dose range the response is sublinear; for ^60^Co gamma irradiation doses from 0.2- to 1 kGy, a trend towards supralinearity is obtained. Fig 5(b) points to substantial trap filling, the glow curves indicating greater propensity towards deeper trap filling (with a shift towards greater temperatures). Fig 5(c) indicates further accessing of deeper traps and finally, at 1 kGy, evidence of growth in trap creation is seen, resulting from irradiation damage.

**Fig 5:** Linearity index function against dose for (a) X-ray irradiation; (b) and (c) refer to gamma irradiation responses in the low dose (2- to 10 Gy) and high dose (0.2- to 1 kGy) regimes.

### 3.3. Energy response

The mass energy absorption coefficients are dependent on the mediating energy-loss processes, including the photoelectric interaction (predominating for low energy x- and gamma-rays (up to several hundred keV), Compton scattering (important at intermediate energies) and pair production (for photon energies ≥ 2m_o_c^2^, where m_o_ is the rest mass and c the speed of light). The probability of each interaction depends not only on the energy of the incident radiation but also on the atomic number (Z) of the irradiated material [12], greatest for the photoelectric effect. Calibration of the dosimetry system is usually obtained for a specified radiation beam quality, Q [20], Q(E) correcting for use at other energies [21]. While in ideal situations the calibration would be independent of energy, in reality determination of Q for a number of radiation measurements is necessary.

To obtain the energy dependence, the borosilicate glass slide dosimeters were irradiated to x-rays generated at nominal potentials of 40, 60, 80, 100, 120, and 140 kVp, each at a fixed dose of 2 Gy. The data obtained were the average of three measurements taken for each sample. Due to the polyenergetic nature of x-ray beams, it is typical for the effective energy to be taken to be either one-third or one-half of the kVp values, providing a measure of mean energy [22]. Using the one-half estimate, the effective energy delivered by 40, 60, 80, 100, 120, and 140 kVp X-rays would be 20, 30, 40, 50, 60 and 70 keV respectively. Fig 6 demonstrates the greatest TL response of the glass slide dosimeters to be at an effective energy (E_eff_) of 60 keV, equating with the diagnostically favourable potential of 120 kVp, dominant energy deposition being via photoelectric interactions [23]. For E_eff_ values progressively below 60 keV the influence of attenuation is increasingly evident, while for E_eff_ above 60 keV the increase in transmission is seen to progressively decrease detection efficiency.

**Fig 6:** Energy response of borosilicate glass slide samples irradiated to a dose of 2 Gy, use being made of x-ray beams of effective energies in the range 20 to 70 keV; also included are ^60^Co gamma irradiations (mean energy 1250 keV). The x-axis is non-linear in order to accommodate the latter.

### 3.4. Glow curve analysis

In order to determine the stability of the TL material for dosimetry, the most important physical factor is the temperature at which the peak of the glow curve occurs [24]. The type and amount of impurities, lattice defects in the material as well as thermal history and treatment of the material will affect the shape of glow curve. The number of traps, both for electrons and holes and hence the amount of charge involved in the transition of electrons from conduction band to the trap center are related with the area under each glow peak. The dosimetric traps require somewhat more energy to release the more deeply trapped electrons, these normally forming the dosimetric peak within which the maximum TL yield is obtained and hence used as the principal peak in dosimetric evaluation.

Fig 7 shows borosilicate glass slide glow curves for x- and gamma radiations, readout being obtained at a heating ramp-rate of 25 °C s^-1^. The full-width at half maximum (FWHM) TL intensity for each dose, from 2- to 10 Gy, are listed in Table 1; the peak width values correspond to the temperature range around which greatest intensity is found. Using GlowView software, a simplified numerical method for background subtraction has been implemented [25]. The borosilicate glass slides glow curves consist of one broad peak, Fig 7 being constructed with the aid of the WinREMs application.

**Fig 7:** Borosilicate glass sample TL glow curves using: (a) 120 kVp x-rays for doses 2–10 Gy; (b) ^60^Co gamma doses from 2–10 Gy and; (c) ^60^Co gamma doses from 0.2–1 kGy.

**Table 1:** Glow curve FWHM (°C) for borosilicate glass irradiated to a range of absorbed dose.

Dose (Gy)	FWHM (°C)		Dose (Gy)	FWHM (°C)
	120 kVp x-rays	^60^Co gamma-rays		^60^Co gamma-rays
**2**	90.0	90	**200**	129.
**4**	99.7	104	**400**	123
**6**	116.3	105	**600**	113
**8**	120.0	103	**800**	117
**10**	121.3	111	**1000**	135

For the 2 to 10 Gy dose range, the glass slide glow curves are seen to cover the overall nominal temperature range 75 to 325 °C, albeit with notable upper temperature restriction applying for doses < 10 Gy. For the 0.2- to 1 kGy gamma irradiations the range extends to 350 °C for all doses, an indicator of deep trap filling and potential deep traps creation. These values accord with the well-established understanding that preferential trap filling occurs, from the filling of the more superficial traps at low dose to deeper traps at greater dose. As an example, across the two gamma dose regimes, 2 to 10 Gy and 0.2 to 1 kGy, a clear shift in peak position towards greater temperatures is observed (Fig 7), linking with the discussion in section 3.2, regarding the Linearity Index. To add emphasis to our earlier discussion on trap stability, in the 2–10 Gy dose regimes, a shift in the temperature for gamma irradiations is apparent in making comparison between these results and those for the X-ray source, which is due to the release of more trapped charged carriers. This increment in TL temperature continues until the point at which the number of trapped electrons in the metastable state is sufficiently depleted and then the TL intensity reduces.

Glow curves deconvolution (Fig 8), based on the first-order kinetics model of Randall and Wilkins (1945) [26], has been carried out aided by GlowFit software. This includes a linear heating profile and glow curve fitting carried out using an iterative Levenberg–Marquardt algorithm. The GlowFit program and its performance has been described in detail by Pulchalska and Bilski (2006) [27], advantageous in analyzing complex glow curves with overlapping peaks. In order to better control the fitting peak parameters, the original algorithm [28, 29] was modified. The area, position (Tm) and height of the glow peak depend on intrinsic parameters such as activation energy (trap depth (E)), frequency factor (s) and concentration of traps, all of these are strongly impressible by fabrication process, and extrinsic ones such as heating rate (β) and absorbed dose [30]. Mentioned trap parameters can be derived from the respective glow curves. Each maximum glow peak comes out from a trapping level and each activation energy could be indicative of a defect type.

**Fig 8:** Deconvolution of the glow curves of borosilicate glass slide dosimeters; (a) refers to irradiations using x-rays generated at an accelerating potential of 120 kVp, for a dose of 10 Gy; (b) and (c) refer to irradiations to ^60^Co gamma for doses of 10 Gy and 1 kGy respectively.

Clark (2012) [12], previously mentioned, investigated commercial borosilicate glass of composition similar to commercial borosilicate containers, obtaining a narrow low-temperature peak and a broad high temperature peak. The number and approximate position of particular deconvolved TL peaks were obtained using the T_max_-T_stop_ method [31], resulting in five peaks in all, centred at approximately 120, 160, 225, 300, and 340°C. Similar investigation conducted by this group on the present material, obtained five peaks, centred at approximately 163, 216, 232, 261 and 278 °C [32]. The plot can also be used to gain an estimate of the kinetics of the electron-hole recombination processes. According to Horowitz et al., (1999) [31] T_max_-T_stop_ is conducted by heating the irradiated sample at a linear heating rate to a temperature (T_stop_) in the low tail of the irradiation peak. The sample is then cooled to room temperature and reheated at the same linear heating rate prior to obtaining the residual intensity. The maximum peak temperature (T_max_) in the glow curve is recorded. The entire process is repeated on a newly irradiated sample with 5 °C increments in T_stop_. Fig 8(a) to 8(c) shows the broad glow curves, optimally consisting of five peaks, with figures of merit (FOM) of between 0.65 to 1.10. The deconvolved glow curves have been evaluated in terms of maximum intensity (I_m_), E, FWHM and peak integral (PI), all tabulated in Table 2. The peak integral, the area under the peak, indicates the number of free electrons transiting from traps to the luminescence centre. The area was found to be highly dependent on dose, as previously discussed. Also of note is that, as E increases the glow peak shifts to higher temperature with a decrease in peak height and increase in width keeping the area constant [33].

**Table 2:** Details of T_m_, I_m_, E, FWHM, PI and s for each peak in the overall glow curve.

**Dose (Gy)**	**Peak**	**T**_**m**_ **(°C)**	**I**_**m**_	**Activation Energy, E (eV)**	**FWHM (°C)**	**Peak Integral (PI)**	**Frequency Factor, s (s**^**-1**^**)**
**10 (X-ray)**	1	153.1	247	0.70	51.0	8.19 ×10^3^	2.23 x 10^8^
	2	181.8	642	0.66	61.1	2.54 ×10^4^	2.02 x 10^7^
	3	216.9	1.23 ×10^3^	0.67	69.8	5.57 ×10^4^	6.35 x 10^6^
	4	256.2	1.04 ×10^3^	0.90	61.7	4.18 ×10^4^	3.16 × 10^8^
	5	294.1	288	1.43	45.4	8.48 ×10^3^	6.32 × 10^12^
**Dose (Gy)**	**Peak**	**T**_**m**_ **(°C)**	**I**_**m**_	**E(eV)**	**FWHM (°C)**	**Peak Integral (PI)**	**Frequency Factor, s (s**^**-1**^**)**
**10 (Gamma)**	1	177.9	42.1	0.81	49.9	1.37 ×10^3^	1.41 × 10^10^
	2	207.8	116	0.77	59.5	4.49 ×10^3^	1.13 × 10^9^
	3	242.3	249	0.80	65.1	1.05 ×10^4^	6.93 × 10^8^
	4	281.2	167	1.26	48.9	5.35 ×10^3^	3.96 × 10^12^
	5	309.4	43.8	2.89	24.2	7.01 ×10^2^	2.75 × 10^26^
**Dose (Gy)**	**Peak**	**T**_**m**_ **(°C)**	**I**_**m**_	**E(eV)**	**FWHM (°C)**	**Peak Integral (PI)**	**Frequency Factor, s (s**^**-1**^**)**
**1000 (Gamma)**	1	185.4	1.43 ×10^4^	0.86	48.8	4.56 ×10^5^	2.98 × 10^9^
	2	213.6	3.00 ×10^4^	0.78	59.9	1.17 ×10^6^	1.10 × 10^8^
	3	254.9	5.53 ×10^4^	0.79	68.8	2.47 ×10^6^	3.15 × 10^7^
	4	297.9	4.38 ×10^4^	1.1	59.7	1.70 ×10^6^	3.68 × 10^9^
	5	333.4	9.79 ×10^3^	2.9	26.1	1.66 ×10^5^	3.08 × 10^24^

Fig 9, obtained from photoluminescence spectroscopy, shows the absorption and emission spectra of the B_2_O_3_ glass slides resulting from exposure to x-rays, providing two main absorption and emission peaks within the range 400 to 1500 nm^-1^ indicated by the first and second peaks, respectively. Residing in the visible region (400–800 nm^-1^), the induced bands are due to positive hole centres from the borate glass matrix and are linked to the generation of either non-bridging oxygen hole centres (NBOHC) or boron oxygen hole centres (BOHC) as previously suggested by Bishay [34] and Friebele [35]. The emissions appearing in the region 900–1400 nm^-1^, residing in the near infrared region, are related to the B-O band stretching vibrations of BO_4_ tetrahedra. Finally, the intense 701 nm^-1^ peak is due to the bending of B-O-B linkages. As expected, ionising radiation causes clear changes in the optical spectra through the capturing and release of pairs of electrons and positive holes as well as the formation of induced defects that reduce the absorption and emission intensity.

**Fig 9:** Emission spectra of borosilicate glass subjected to x-ray doses of 0, 6 and 10 Gy, use being made of a Photoluminescence (PL) system with a 40 × objective lens and stimulation by a laser at 325 nm. The grating system offers 1200 lines/mm and the PL intensity is detected using a CCD camera of 578 × 400 pixels.

Electron paramagnetic resonance (EPR) analysis has been undertaken by Clark (2012) on commercial borosilicate glass; results showed production of boron oxygen hole centre (BOHCs) and E′-defect centres (network defects), suggesting that the BOHC is involved in the recombination process occurring during TL measurement where it is likely that trapped electrons recombine with trapped BOHC. EPR results for the different borosilicate glasses also showed that approximately the same number of BOHC are created per dose regardless of the glass source. This means that the formation of BOHC alone cannot explain the different response in the overall intensity of the TL glow curves in borosilicate glass from different regions.

### 3.5. Fading

McKeever et. al (1995) [17] and Rivera (2012) [36] have described fading as the loss of signal or decrease of post-irradiation TL yield over a period of time prior to TL readout, a period within which the more low-lying traps are partially emptied. This can happen either through thermal or optical excitation of trapped electrons, or both. Even at significantly lower temperature than the glow peak temperature of a particular TL material, thermal fading can still take place due to the quantum tunnelling effect, the mean lifetime of electrons in shallow traps being very short [37]. The parameters that govern the rate of thermal fading are the trap depth, E, and the frequency factor, s. A combination of a low value of E and a high value of s can be expected to produce TL material with a higher fading rate than the converse situation.

In regard to the above, there is a need to detail the loss of TL response post irradiation. In present work, study has been made of the TL-signal lost by the borosilicate glass slide dosimeters x-ray irradiated to doses from 2 to 10 Gy. For this, use has been made of the X-ray source operated at a potential of 120 kVp, fading being studied for different delay periods, up to a maximum of 35 days (Table 3 shows the percentage residual signal). From Fig 10(a), it is apparent that some 54%, 51%, 51%, 54% and 42% of the signal are lost within the 35 days period for 10, 8, 6, 4 and 2 Gy doses, respectively. As such, it is clear that a useable signal is retained for in excess of a calendar month. As can be seen in Fig 10(b), a rapid decrease in signal intensity is observed during the first 24 hours post irradiation, giving a mean loss of TL response for the glass slide sample of some 0.7% per hour, with a decay factor of -13.8. However, the radiation response requires correction factors for improved accuracy, accounting for various influencing factors, including sensitivity to dose, energy dependence and fading.

**Fig 10:** The loss of TL yield of borosilicate glass slides over a period of (a) 35 days post-irradiation for x-ray doses from 2 to 10 Gy and (b) within 24 hours post-irradiation subjected to an x-ray dose of 2 Gy.

**Table 3:** Residual signal (%) of borosilicate glass slides for doses from 2 to 10 Gy irradiated with 120 kVp X-rays within 35 days of evaluation.

Dose (Gy)	Number of Days Post Irradiation	1	7	14	21	28	35
**2**	**Residual Signal (%)**	100	70.4	67.8	61.4	54.8	48.9
**4**		100	61.7	51.8	49.9	46.9	46.2
**6**		100	60.5	50.5	46.8	45.9	44.5
**8**		100	60.8	52.4	52.2	47.7	46.7
**10**		100	56.2	49.1	47.1	46.6	45.1

### 3.6. Elemental analysis and effective atomic number, Z_eff_

An energy dispersive X-ray analyzer (EDX) attached to a scanning electron microscope (SEM) was used for further characterization of the borosilicate glass slides. The presence of boron in the structure of silica glass slide was confirmed, also showing good uniformity of distribution of silicon, oxygen, sodium, carbon, calcium, magnesium and aluminium in the glass slide structure (see Table 4). The average EDX measured boron concentration from three scanned spots was found to be 6.5%.

**Table 4:** Elemental composition of borosilicate glass slides, obtaining from EDX measurement.

Elements	Average Fractional Weight (W_i_) for each element
**oxygen, O**	0.5233
**silica, Si**	0.2122
**boron, B**	0.1066
**sodium, Na**	0.0656
**potassium, K**	0.0844
**calcium, Ca**	0.0179
**titanium, Ti**	0.0058
**aluminium, Al**	0.0004
**magnesium, Mg**	0.0003

Extending out of this is one of the most convenient parameters representing radiation interactions within the medium, namely the effective atomic number, Z_eff_. This can be defined as a weighted arithmetic mean of the atomic number of the constituent atoms [38] and can be calculated using the Mayneord equation as shown below:

$${\text{Z}}_{\text{eff}}={\left({\text{a}}_{1}{\text{z}}_{1}{}^{\text{m}}+{\text{a}}_{2}{\text{z}}_{2}{}^{\text{m}}+{\text{a}}_{3}{\text{z}}_{3}{}^{}+\ldots \ldots {\text{a}}_{\text{n}}{\text{z}}_{\text{n}}{}^{\text{m}}\right)}^{1/\text{m}}$$ (3)

where a_1_, a_2_…a_n_, are the fractional contributions of each element to the total number of electrons in the mixture and m is equal to 2.94 (an index reflecting the Z-dependence of photon energies in the photoelectric dominated region below some 100 keV). By using elemental fractions of the samples obtained by EDX analysis in Eq 3, Z_eff_ for borosilicate glass slide samples has been found to be 11.9, not greatly dissimilar to the effective atomic number of Ge-doped fibres [39] of 12.2, also within the bounds of the effective number of bone (in the range 11.6–13.8). As such, a particular application foreseen for the borosilicate glass slide samples would be in bone dosimetry. Dosimetric utilisation of commercial borosilicate glass as a new dosimeter has previously been reported by members of this group, evidence being shown of the mass-energy absorption coefficients for borosilicate glass. More generally they are seen to better match to that of NIST B-100 Bone Equivalent Plastic (being of relatively large Z_eff_). However, from 50 keV up to 100 keV the reduced energy dependent Compton scattering dominates, the borosilicate glass then trending towards closer accord with lower Z_eff_ media such as soft tissues [40].

## 4. Conclusion

Present investigation has evaluated a range of TL and other dosimetric properties for commercial borosilicate (B_2_O_3_) glass slides, including dose response, sensitivity, repeatability, energy response, fading and glow curves, for x- and gamma- rays doses, 2 Gy to 1 kGy. For x-ray doses from 2 to 10 Gy the sensitivity has been found to be some 5 times that of the equivalent doses of ^60^Co gamma irradiations, indicative of the population of specific electron/hole traps differing with the type of ionizing photon radiation. The borosilicate glass slides offer repeatable response to within 1% in respect of x-ray irradiation. Analysis of the linearity index showed the x- and gamma responses in the low dose regime exhibiting similar patterns, growing in a sublinear fashion as dose is increased. In contrast, at high gamma dose, 0.2–1 kGy, the linearity index provides a supralinear response with increase in dose. The energy response has indicated suitability of the proposed materials for use as radiation dosimeters in clinical radiation therapy, also perhaps not excluding use in high dose clinical x-ray angiographic procedures. There are two main separate broad absorption and emission bands in the spectral regions 400–800 and 900–1400 cm^-1^ respectively, as observed in photoluminescence spectra, noting changes in the optical spectra through the capturing and release of pairs of electrons and positive holes. Building up from this, deconvolution of glow curve showed five underlying peaks. In particular, the measurements yield information on the activation energy, E (eV) and the frequency factor, s (s^-1^). Summarily, the TL sensitivity of the studied samples depends on its physical form, impurity, type and energy of the ionizing radiation and readout system used (heating rate). Finally, issues such as the non soft-tissue equivalence of the dosimeter and TL decay rate require correction factors to be applied in order to minimize errors in determination of dose.
